The article "Deep Learning-Based Correlation Analysis between the Evaluation Score of English Teaching Quality and the Knowledge Points" was published in 2022. Journal: Comput Intell Neurosci.

# Deep Learning-Based Correlation Analysis between the Evaluation Score of English Teaching Quality and the Knowledge Points

**DOI:** 10.1155/2022/4102959

**Published:** 2022-08-25

**Authors:** Yuanyuan Li

**Affiliations:** Foreign Language School, Suzhou Vocational University, Suzhou 215104, China

## Abstract

As one of the three main courses from primary school to senior high school, improving the quality of English teaching in and out of class has become the top priority of colleges and universities. English knowledge points are complex, and domestic scholars have studied vocabulary knowledge and grammatical awareness from various perspectives, but there is still a lack of research on the correlation between vocabulary knowledge, grammatical awareness, and cloze test scores of senior high school students. Therefore, this paper carries out empirical research from the depth of English vocabulary, English grammar, reading comprehension, cloze test, and composition, aiming at exploring the relationship between teaching quality and English knowledge points. Classroom teaching quality evaluation is the basic content of education quality evaluation, which not only needs to evaluate the effect of class hours but also needs a student's long-term learning effect. In order to improve the quality of classroom English teaching, enrich the content of classroom English, and ultimately make the quality of students' learning to a higher level, the combination model of the teaching quality evaluation index is established by combining the decision tree with the knowledge point rule association method and the evaluation results are verified by association rule analysis. This paper selects the effective indicators that affect the evaluation of English teaching quality, determines the weight of the indicators by using the analytic hierarchy process, effectively constructs the combination model of the decision tree and rule association method, and establishes the evaluation model of students' English learning ability in the classroom. Taking students as the main object and combining them with the requirements of digital teaching, the evaluation index system is formed, the index weight is determined by using the analytic hierarchy process, and the classroom teaching quality evaluation model based on the decision tree and English knowledge point correlation analysis is constructed to truly reflect the teaching level of teachers, and the correlation analysis is carried out between English teachers' own quality and students' learning effects and knowledge points. By testing the model performance of English vocabulary depth, reading comprehension, grammar, writing, and other knowledge points, we can well evaluate and analyze students' mastery of English learning and the correlation of English knowledge points.

The article "Deep Learning-Based Correlation Analysis between the Evaluation Score of English Teaching Quality and the Knowledge Points" was published in 2022. Journal: Comput Intell Neurosci.

## 1. Introduction

English is the most common language in the world, and its importance goes without saying. In order to evaluate the quality of English teaching in schools and study the correlation between teaching quality and English knowledge points, we have constructed a combined evaluation system of the decision tree and rule association analysis of knowledge points. This paper expounds that this method is efficient in detecting large error data in fringe images [1] and uses artificial intelligence technology to evaluate the quality of surgery in medicine [2]. It expounds the anatomical analysis of the components of kidney stones by the deep learning method [3]. In order for the leaders of colleges and universities to do a better job in teaching management and reduce unnecessary management problems, literature [4] fully demonstrates the effectiveness of teaching evaluation for students in colleges and universities under the background of intelligent computing. Using big data related knowledge to study the evaluation system of college physical education can not only promote the implementation of college physical education evaluation but also effectively improve the quality of college physical education [5]. It takes the quality of graduates as the core content, establishes a result-oriented evaluation system of teaching quality in colleges and universities, and finds that the academic level and the level of competition in choosing jobs are two quantitative levels reflecting the quality of graduates [6]. It mainly puts forward some measures to construct the evaluation system of college English teaching from the key point of constructing the evaluation system of junior and senior high school English teaching based on online learning platform [7]. Through a scientific and complete teaching evaluation system, we can optimize the physical education teaching process to a certain extent, promote the effective realization of physical education teaching objectives, and improve the quality and efficiency of physical education in colleges and universities [8]. It expounds the development of task-based learning as the center of the English teaching evaluation model and cultivates the English writing ability and creative thinking of Thai sixth grade students [9]. It mainly explores the multidimensional teaching evaluation system of local universities under the background of transformation [10]. It discusses how higher education institutions apply the questionnaires used in our research to diversity management [11]. It implements gauge teaching evaluation from the perspective of students and teachers [12]. There are considerable problems in the hypothesis of students' evaluation to measure the teaching effect, especially in the system where problem-based learning is the main teaching idea. It determines a working hypothesis; that is, students do not use teaching ideas as the main motivation to evaluate employees, which leads to an abnormal incentive [13]. This study assessed the effectiveness of focused educational practice designed for teachers in multiple professional departments, which have a large number of elderly patients, and became a geriatrics-based teacher development plan [14]. This paper explores the diversity of evaluation methods and exerts the positive functions of evaluation, detection, stimulation, and development. By expanding evaluation ideas, emphasizing performance evaluation, realizing immediate evaluation, and carrying out special evaluation, the evaluation function can be repositioned [15]. The paper verifies the effectiveness and practicability of our method through an intuitive multimedia teaching evaluation example [16]. The analysis results of this paper may provide some theoretical basis and reference for the research of history teaching methods and also provide relevant information for overseas Chinese modern history research institutions to understand the learning situation of Chinese history in this period [17]. On the basis of continuous development and improvement of teaching evaluation, this paper explores the refined management of undergraduate teaching [18]. Teaching evaluation is an important part of curriculum teaching, which is beneficial for teachers to get feedback, improve the teaching quality, and maintain the teaching foundation. It is an effective measure for students to find the most suitable learning method, correct learning habits, and improve learning efficiency [19]. The fuzzy comprehensive evaluation of the cloud system is studied, and finally the experimental verification is carried out by an example [20]. The purpose of this study is to analyze the relationship between learning styles and academic achievements of accounting science students combined with teachers' evaluation [21]. It examines the evaluation degree of teachers' own teaching behavior management practice, as measured by the evaluation system of classroom learning strategies [22]. The teaching evaluation method proposed in this study is helpful to fully reflect the quality of classroom teaching and guide students' professional development [23]. In this paper, we propose two vocabulary-based methods, especially knowledge-based and machine learning-based methods, to automatically extract opinions from short comments [24]. This structured process produces an evidence-based and systematically developed EM teacher evaluation tool, which can provide teachers with real-time operational feedback and support improved clinical teaching [25].

The article "Deep Learning-Based Correlation Analysis between the Evaluation Score of English Teaching Quality and the Knowledge Points" was published in 2022. Journal: Comput Intell Neurosci.

## 2. Construction of the Index System of the English Teaching Quality Evaluation Model

### 2.1. Indicator Construction

The evaluation of English teaching quality from primary school to senior high school is a nonstatic process involving many variables and influencing factors. The evaluation system of English teachers' classroom teaching quality needs to reflect and exclude teachers' own influencing factors, such as teachers' teaching concepts, teaching attitudes, teaching methods, and educational effects. It is also necessary to take into account the factors of students who directly participate in teaching. Students can directly feel teachers' own teaching quality and students' learning effects during the whole feeling process of participating in classroom teaching. The innovation and diversification of information-based foreign language teaching methods require the cultivation of students' intrinsic motivation and self-efficacy and the effective integration of information technology and foreign language teaching. Finally, it establishes the initial index content composed of four most important indexes and fifteen more important indexes: “curriculum goal, classroom teaching, teaching effect, and teaching expansion.”

1. The index of “curriculum goal” is the direction and soul of the curriculum, which determines the overall quality of personnel training. It aims to reflect the applicability of teaching content and cultivates the matching degree of knowledge and skills that students need to achieve through curriculum study.
2. The index of “classroom teaching” reflects the main forms and key links of English teaching from primary school to senior high school, including the effectiveness of English classroom teaching activities in cultivating knowledge depth and learning ability, the rationality of classroom teaching time and content arrangement, and the breadth and depth of information resources use under the background and environment of the digital age.
3. The “Teaching effect” reflects the effectiveness measurement index after the teaching process, especially reflects the advancement of foreign language teaching supported by information technology and its promotion to the teaching effect.
4. “Teaching expansion” refers to the teaching methods outside the classroom, which are carried out around the curriculum objectives under the support of information technology. The design and effect evaluation of extracurricular learning content to assist classroom teaching and enrich related courses, including the diversification of extracurricular learning resources and assessment contents and methods, the abundance of resources provided online and offline, and the effectiveness of promoting college English learning.

The article "Deep Learning-Based Correlation Analysis between the Evaluation Score of English Teaching Quality and the Knowledge Points" was published in 2022. Journal: Comput Intell Neurosci.

### 2.2. Teaching Evaluation Process

The evaluation process is the selection of teaching quality and teachers' own quality evaluation indicators from two aspects; one is the relevant data of teachers, and the other is the related factors of teaching schedule and teaching links. Obtain the English teaching evaluation data package from the educational administration platform, initialize the data according to indicators, generate samples to be evaluated, calculate entropy increment values of all indicators to generate a decision tree, and verify the classification rules of English teaching quality evaluation generated by the decision tree by the association rules method. In this, the specific steps for verifying the decision tree and association rule combination model are shown in Figure 1.

## 3. Description of the Algorithm

### 3.1. Decision Tree and Knowledge Point Association

The decision tree is mainly composed of roots, branches, and leaves. The calculation method of expected entropy is as follows:

(1) $$\begin{array}{c} I\left(s_{1},s_{2},s_{3},\ldots ,s_{m}\right)=-\sum_{i=1}^{m}\frac{s_{i}}{s}\log_{2}\frac{s_{i}}{s}. \end{array}$$

Let the expected expression of an attribute *A* of the sample be

(2) $$\begin{array}{c} E\left(A\right)=\sum_{j=1}^{m}\frac{s_{ij}+s_{2j}+\ldots +s_{mj}}{s}I\left(s_{ij},s_{2j}+\ldots +s_{mj}\right). \end{array}$$

For the subset *Is*_*j*_ is defined as follows:

(3) $$\begin{array}{c} I\left(s_{ij},s_{2j}+\ldots +s_{mj}\right)=-\sum_{i=1}^{m}\frac{s_{ij}}{s_{j}}\log_{2}\frac{s_{ij}}{s_{j}}. \end{array}$$

Expected Entropy Gain of *A* to *S* is

(4) $$\begin{array}{c} \text{Gain}\left(A\right)=I\left(s_{ij},s_{2j}+\ldots +s_{mj}\right)-E\left(A\right). \end{array}$$

The gain rate is expressed as

(5) $$\begin{array}{c} \text{Gain}\left(A\right)=\frac{\text{Gain}\left(A\right)}{\text{splitinf}o\left(s\right)},\\ \text{splitinfo}\left(s\right)=\sum_{i=1}^{m}\frac{s_{i}}{\left|s\right|}\times \;\log_{2}\frac{s_{i}}{\left|s\right|}. \end{array}$$

### 3.2. Correlation Analysis of Knowledge Points

Suppose that the number of items in all sets *D* is *D*, *X* is an item set in *D*, and the number of item sets in *D* is count, then the support degree of *X* is

(6) $$\begin{array}{c} \text{support}\left(X\right)=\frac{\text{count}\left(X\subseteq D\right)}{\left|D\right|}. \end{array}$$

Let any two item sets *X* and *Y* in *D* satisfy the condition *X* ⊂ *D*, *Y* ⊂ *D*, they are independent of each other, and the probability that they appear at the same time in *D* can also be expressed by support:

(7) $$\begin{array}{c} \text{support}\left(X\Rightarrow Y\right)=\frac{\text{count}\left(X\cap Y\right)}{\left|D\right|}. \end{array}$$

In addition to calculating support, reliability can also be used to measure the relationship between *X* and *Y*:

(8) $$\begin{array}{c} \text{confidence}\left(X\Rightarrow Y\right)=\frac{\text{support}\left(X\Rightarrow Y\right)}{\text{support}\left(X\right)}. \end{array}$$

It can also be measured by the degree of improvement:

(9) $$\begin{array}{c} \text{lift}\left(X\Rightarrow Y\right)=\frac{\text{confidence}\left(X\Rightarrow Y\right)}{\text{support}\left(X\right)}. \end{array}$$

The article "Deep Learning-Based Correlation Analysis between the Evaluation Score of English Teaching Quality and the Knowledge Points" was published in 2022. Journal: Comput Intell Neurosci.

### 3.3. RCNet Model

RCNet consists of four parts, namely, the output layer, bidirectional GRU layer, attention layer, and prediction layer. In this, GRU is selected to learn the calculation formula of remote dependency of the whole input sequence as follows:

(10) $$\begin{array}{c} z_{n}=\sigma_{g}\left(w_{z}x_{n},+u_{z}h_{n-1}+b_{z}\right),\\ r_{n}=\sigma_{g}\left(w_{r}x_{n},+u_{r}h_{n-1}+b_{r}\right),\\ {\hat{h}}_{n}=\emptyset_{h}\left(w_{h}x_{n},+u_{h}\left(r_{n}*h_{n-1}+b_{h}\right),\right.\\ GRU\left(h_{n-1},x_{n}\right)=\left(1-z_{n}\right)*h_{t-1}+z_{n}*{\hat{h}}_{n}. \end{array}$$

The hidden layer vector of the bidirectional GRU is calculated as follows:

(11) $$\begin{array}{c} \overset{⟶}{h_{n}}=GRU\left(\overset{⟶}{h_{n-1}},x_{n}\right),\\ \overset{⟶}{h_{n}}=GRU\left(\overset{\leftarrow }{h_{\left.n-1\right)}},x_{n}\right),\\ h_{n}=\left[\overset{⟶}{h_{n}},\overset{\leftarrow }{h_{n}}\right]. \end{array}$$

The *N* word vectors are fused into

(12) $$\begin{array}{c} \bar{Q_{i}}=\text{avg}\left(h_{1},h_{2},\text{…},h_{N}\right)\in R^{2u}. \end{array}$$

In the further calculation, the influence of TC and TQ tail is eliminated by the mask method, namely,

(13) $$\begin{array}{c} G\left(i,j\right)=\left\{\begin{array}{cc} H_{C}{\left(i\right)}^{T}H_{Q}\left(j\right), & i<\left|TC\right|,<\left|TQ\right|\\ 0, & i\geq \left|TC\right|or\;j\geq \left|TQ\right|. \end{array}\right. \end{array}$$

After obtaining the paired matching matrix, the attention layer applies the softmax function to each column in *G* to obtain the probability distribution of each column, wherein when considering a single test word, each column in the matrix represents a separate text-level attention, the text-level attention of the nth word is as follows:

(14) $$\begin{array}{c} a\left(n\right)=\text{soft}\max\left(G\left(1,n\right),\ldots ,G\left(\left|TC\right|,n\right)\right). \end{array}$$

Calculate reverse attention; that is, for words in the nth chapter, calculate the importance distribution of test words to indicate which test words are more important for individual words in the chapter. The attention mechanism will gradually implement the softmax function and apply it to each pair of matching matrices to obtain the attention of English test questions with different difficulties:

(15) $$\begin{array}{c} \beta \left(n\right)=\text{soft}\max\left(G\left(n,1\right)\right),\ldots ,G\left(n,\left|TQ\right|\right). \end{array}$$

Get the average attention at the test level as follows:

(16) $$\begin{array}{c} \beta =\frac{1}{\left|TC\right|}\sum_{N=1}^{\left|TC\right|}\beta \left(n\right). \end{array}$$

Explicitly understand the contribution of each test word, vote according to the importance of each test word, and output the final text-level attention weight as the text-level attention vector as follows:

(17) $$\begin{array}{c} CA_{i}=a^{T}\beta . \end{array}$$

The expression for predicting the difficulty of English test questions is as follows:

(18) $$\begin{array}{c} \tilde{P}=\text{Sigmoid}\left(W_{2},o_{i},+b_{2}\right). \end{array}$$

Training model expression is as follows:

(19) $$\begin{array}{c} J\left(\theta \right)=\sum_{T_{t},Q_{i},Q_{j}}{\left(\left(P_{i}^{t}-P_{j}^{t}\right)-\left(\tilde{P_{i}^{t}}-\tilde{P_{j}^{t}}\right)\right)}^{2}+\lambda_{\theta }\theta_{M}^{2},\\ \text{RMSE}=\sqrt{\frac{1}{m_{i}}\sum_{j=1}^{m_{i}}{\left(P_{ij}-\tilde{R_{ij}}\right)}^{2}},\\ R^{2}=1-\frac{\sum_{j=1}^{m_{i}}{\left(P_{ij}-\tilde{R_{ij}}\right)}^{2}}{\sum_{j=1}^{m_{i}}{\left(R_{i}-\tilde{R_{ij}}\right)}^{2}}. \end{array}$$

The article "Deep Learning-Based Correlation Analysis between the Evaluation Score of English Teaching Quality and the Knowledge Points" was published in 2022. Journal: Comput Intell Neurosci.

## 4. Experiment

### 4.1. Simulation Experiment

#### 4.1.1. Data Set Introduction

The sample data set adopted in this experiment is the English test results and answer records from many middle schools in China from 2014 to 2021. Each data include five fields: English test content, question, correct option, wrong option, and test difficulty. The statistical results are shown in Table 1.

The difficulty of the experimental data set is tested, and the uniformity of the difficulty distribution of the test questions is distributed by the classical measurement theory difficulty of 0–1, as shown in Figure 2.

### 4.2. Experimental Research

The correlation between the quality of English teaching and the breadth and depth of vocabulary is analyzed. This question verifies the correlation between English teaching quality, vocabulary breadth knowledge, and vocabulary depth knowledge. It is necessary to check whether there are singular values in the whole data so as to analyze whether there is a curve relationship between the data. Therefore, before testing the correlation coefficient, we draw scatter charts on the relationship between the teaching quality of English learning and vocabulary breadth knowledge and vocabulary depth knowledge as shown in Figure 3.

The article "Deep Learning-Based Correlation Analysis between the Evaluation Score of English Teaching Quality and the Knowledge Points" was published in 2022. Journal: Comput Intell Neurosci.

The effectiveness of the index system of the traditional English classroom teaching quality evaluation model is to ensure students' trust in the evaluation results of college English classroom teaching quality. The purpose of training the students before the evaluation is to let them know the purpose and significance of the evaluation and to guide students to deepen their familiarity with the indicators and grading standards. Finally, the scoring results are collected, and according to the students' scoring data, the actual scores of teaching quality evaluation are calculated. The results are shown in Table 2.

The above data are counted into tables as shown in Figure 4.

### 4.3. Model Comparison

For English learning vocabulary depth, grammar, reading comprehension, cloze, writing, and other knowledge points, student-centered teaching quality evaluation uses their mastery to evaluate teachers' English teaching quality. Based on the above index standards, we use the decision tree method under deep learning to study and evaluate English teaching quality evaluation. The experimental data are given in Table 3.

Three senior high school students were selected to evaluate the teaching ability, teaching attitude, teaching content, teaching methods, and teaching effect of English teachers as the quality indicators of English classroom teaching and to evaluate the quality of each English learning knowledge point.

The combination model of the decision tree and knowledge point association rule mining is used to evaluate the teaching quality of English vocabulary depth, as shown in Figure 5.

The combination model of the decision tree and knowledge point association rule mining is used to evaluate the teaching quality of English grammar, as shown in Figure 6.

The combination model of the decision tree and knowledge point association rule mining is used to evaluate the teaching quality of English reading comprehension, as shown in Figure 7.

The combination model of the decision tree and knowledge point association rule mining is used to evaluate the teaching quality of the English cloze test, as shown in Figure 8.

The combination model of the decision tree and knowledge point association rule mining is used to evaluate the teaching quality of English writing ability as shown in Figure 9.

### 4.4. Contrast Experiment

The decision tree model and rule mining association combination model proposed in this paper are tested in terms of model performance, and different English knowledge points are compared, as shown in Table 4.

The article "Deep Learning-Based Correlation Analysis between the Evaluation Score of English Teaching Quality and the Knowledge Points" was published in 2022. Journal: Comput Intell Neurosci.

The comparison table between teaching quality and English knowledge points is counted into a bar chart, as shown in Figure 10.

## 5. Conclusion

We analyze the relationship between the effective evaluation of teaching quality in the college English classroom and knowledge points and propose a combined model based on the decision tree and rule association analysis of English knowledge points to evaluate teaching quality in English classrooms. Through the combination model of the two methods to evaluate the teaching quality in the classroom, the evaluation results of teaching quality after evaluation are obtained, which shows that this method is effective and has strong applicable value for the evaluation of English teaching quality in the classroom. The results are as follows:

1. In the difficulty test of English, the difficulty distribution of test questions is relatively uniform. In the difficulty interval of classical measurement theory from 0 to 1, the proportion of test questions in each difficulty interval with a difficulty interval of 0.1 is about 10%.
2. By comparing the actual values of different weights of English teaching indicators with the evaluation values, we can see that the evaluation performance of this model is good.
3. The limitations of the decision tree model combined with rule association analysis can greatly improve the evaluation level of English teaching quality inside and outside the classroom and study and analyze the relevance of English knowledge points.

## Figures and Tables

**Figure 1:** Evaluation process.

**Figure 2:** Difficulty distribution of test questions.

**Figure 3:** Scatter plot of English learning quality and vocabulary breadth knowledge level.

**Figure 4:** Comparison between the actual value and the evaluation value.

**Figure 5:** Comparison of vocabulary depth teaching quality.

**Figure 6:** Comparison of grammar teaching quality.

**Figure 7:** Comparison chart of reading comprehension teaching quality.

**Figure 8:** Comparison of cloze teaching quality.

**Figure 9:** Comparison of English writing teaching quality.

**Figure 10:** Comparison between teaching quality and English knowledge points.

**Table 1:** Quantitative statistics of text length.

Statistical parameters	Quantity
Content and text length of English test questions	53003
Length of English text	11393
Length of question text	3291
Length of option text	9132

**Table 2:** The actual value and evaluation value of teaching quality evaluation.

Weight	Evaluation value	Actual value
K11	0.78	0.69
K12	0.82	0.80
K32	0.81	0.83
K31	0.79	0.87
K35	0.88	0.89
K41	0.83	0.88
K43	0.91	0.90

The article "Deep Learning-Based Correlation Analysis between the Evaluation Score of English Teaching Quality and the Knowledge Points" was published in 2022. Journal: Comput Intell Neurosci.

**Table 3:** Comparison of learning effects of knowledge points.

Category of knowledge points	Learning effect (%)	Teaching effect (%)
Vocabulary depth	82	82
Grammar	88	76
Reading comprehension	79	79
Cloze	78	80
Writing	82	83

**Table 4:** Performance comparison of knowledge points.

Category of knowledge points	Accuracy	Precision	Recall	F1	AUC
Vocabulary depth	0.813	0.861	0.891	0.791	0.815
Grammar	0.824	0.854	0.882	0.832	0.824
Cloze	0.841	0.860	0.883	0.814	0.803
Reading comprehension	0.852	0.866	0.873	0.853	0.815
Writing	0.887	0.871	0.838	0.856	0.887

## Data Availability

The experimental data used to support the findings of this study are available from the corresponding author upon request.
